# Improving Small Intestinal Motility in Experimental Acute Necrotising Pancreatitis by Modulating the CPI-17/MLCP Pathway Using Chaiqin Chengqi Decoction

This article has been retracted.

**DOI:** 10.1155/2020/9189457

**Published:** 2020-02-10

**Authors:** Ziqi Lin, Chenlong Zhang, Xiaoxin Zhang, Na Shi, Yongjian Wen, Chengxia Han, Dan Du, Tingting Liu, Tao Jin, Lihui Deng, Kun Jiang, Xiaonan Yang, Jia Guo, Anthony Philips, Robert Sutton, John A. Windsor, Wei Huang, Ping Xue, Qing Xia

**Affiliations:** ^1^Department of Integrated Traditional Chinese and Western Medicine, Sichuan Provincial Pancreatitis Centre and West China-Liverpool Biomedical Research Centre, West China Hospital, Sichuan University, Chengdu, China; ^2^Department of Traditional Chinese Medicine, Xiang'an Hospital of Xiamen University, School of Medicine, Xiamen University, Xiamen, China; ^3^West China-Washington Mitochondria and Metabolism Centre, West China Hospital, Sichuan University, Chengdu, China; ^4^Applied Surgery and Metabolism Laboratory, School of Biological Sciences, University of Auckland, Auckland, New Zealand; ^5^Liverpool Pancreatitis Research Group, Royal Liverpool University Hospital and Institute of Translational Medicine, University of Liverpool, Liverpool, UK; ^6^Surgical and Translational Research Centre, Faculty of Medical and Health Sciences, University of Auckland, Auckland, New Zealand

## Abstract

Protein kinase C-potentiated inhibitor protein of 17 kDa (CPI-17), a specific inhibitor of myosin light-chain phosphatase (MLCP) regulated by proinflammatory cytokines, is central for calcium sensitisation. We investigated the effects of chaiqin chengqi decoction (CQCQD) on the CPI-17/MLCP pathway in the small intestinal smooth muscle cells (SMCs) and strips (SMS) in an AP model. Necrotising AP was induced in rats by intraperitoneal injections (IPI) of L-ornithine (3.0 g/kg, pH 7.0; hourly × 2) at 1 hour apart; controls received saline. In treatment groups, carbachol (CCh; 60 *μ*g/kg, IPI) or CQCQD (20 g/kg; 2-hourly × 3, intragastric) was administered. The necrotising AP model was associated with systemic inflammation (serum IL-1*β* and TNF-*α*) and worsened jejunum histopathology and motility (serum vasoactive intestinal peptide and intestinal fatty acid-binding protein) as the disease progressed. There was decreased intracellular calcium concentration ([Ca^2+^]_i_) SMCs. Contractile function of isolated SMCs was reduced and associated with down-regulated expression of key mRNAs and proteins of the CPI-17/MLCP pathway as well as increased IL-1*β* and TNF-*α*. CQCQD and CCh significantly reversed these changes and the disease severity. These data suggest that CQCQD can improve intestinal motility by modulating the CPI-17/MLCP pathway in small intestinal smooth muscle during AP.

## 1. Introduction

Gut dysfunction is a common feature of severe acute pancreatitis (AP), although it has yet to be included in any system scoring organ dysfunction severity. Gut dysfunction, often evident as an ileus, is one of the most frequent early complications of AP, and its incidence is higher than respiratory dysfunction [1]. The degree of gut dysfunction is proportionally associated with worsened clinical outcomes of AP [2, 3]. The gut is both a victim and a culprit in acute and critical illness. Intestinal ischaemia [4], decreased gut dysmotility [5], increasing intestinal permeability [6], disruption of mucosal epithelial integrity [7], disruption of intestinal bacterial ecology [8], and impaired mucosal immunity [9] are commonly seen during AP, and the injured gut also amplifies systemic injury and organ failure [10–13].

The mechanisms underlying the development of gut dysmotility are complex. Neural reflexes, hormonal influences, jejunal mitochondrial dysfunction, local molecular inflammatory responses, and the recruitment of activated immune cells into the intestinal muscle are involved [14–17]. It is well documented that proinflammatory cytokines such as interleukin-1beta (IL-1*β*) and tumour necrosis factor-alpha (TNF-*α*), released at the early stage of AP, can further worsen gut dysmotility [18, 19], thus contributing to severe AP development [20]. However, the detailed mechanism of gut dysfunction caused by the inflammatory mediators in AP is still unclear, and few studies have examined the molecular signal transduction pathways in the intestinal smooth muscles.

We have recently shown that gut dysmotility was common in L-arginine-induced necrotising AP in rats and was associated with increased serum vasoactive intestinal peptide (VIP), intestinal fatty acid-binding protein (iFABP) and substance P, indirect parameters of gut injury, and dysmotility. Intragastric administration of chaiqin chengqi decoction (CQCQD), a Chinese herbal formula that is widely used to treat patients with severe AP, decreased pancreatic and gut injury and improved gut motility parameters (serum VIP, iFABP, and substance P). This protective effect was partially via its regulating role of protein kinase C (PKC)-mediated Ca^2+^ release in colonic smooth muscle cells (SMCs) [21]. Since L-arginine at high doses directly induces gut injury and dysmotility by releasing neurotransmitters [21], the effect of CQCQD on improving gut motility needs to be validated in other models of AP induced by toxins that have no direct effect on the gut. Furthermore, emerging evidence has shown that small intestine injury appeared early than colonic injury [12, 14, 22] and was the primary bacterial translation site [23].

The contraction of gut SMCs primarily relies on increase of intracellular calcium concentrations ([Ca^2+^]_i_) and Ca^2+^ sensitivity of myofilaments by elevating phosphorylation of Ser^19^ on the 20-kDa regulatory light chain of myosin II (MLC20) [24]. In the initiate contraction phase, the increased [Ca^2+^]_i_ mediated by the inositol triphosphate receptor activate myosin light-chain kinase (MLCK), a Ca^2+^/calmodulin-dependent enzyme, leading to MLC20 phosphorylation. In the Ca^2+^-independent sustained contraction phase, MLC20 phosphorylation involves inhibition of the myosin light-chain phosphatase (MLCP) pathway which is mediated by the G_*α*q/*α*13_-coupled receptors initiated by sequential activation of G_*α*q/*α*13_, RhoGEF, and RhoA and regulated directly by phosphorylating the myosin-targeting subunit of MLCP (MYPT1) and/or indirectly via the protein kinase C (PKC)-potentiated phosphatase inhibitor of l7 kDa (CPI-17) [25]. CPI-17 is the endogenous heat stable, is a specific inhibitor of MLCP, is central for calcium sensitisation and regulated by proinflammatory cytokines [15, 26, 27], but its role in small intestinal smooth muscles during AP has never been studied.

It is well reported that the contraction function in the gut smooth muscle is strongly linked to the reduced expression of CPI-17 caused by IL-1*β* and TNF-*α* during intestinal inflammation [28–30]. The aim of this study is to investigate the effect of CQCQD on gut injury and dysmotility in a rodent model of L-ornithine-induced necrotising AP and whether this involves modulation of the CPI-17/MLCP pathway.

## 2. Materials and Methods

### 2.1. Animals and Ethics

Male adult Sprague Dawley rats (220–260 g) were purchased from the Experimental Animal Centre of West China Centre of Medical Sciences of Sichuan University (Chengdu, China). The animals were housed in individual cages with free access to water and standard laboratory chow. Housing conditions were kept constant with the temperature at 23 ± 2°C, the relative humidity at 40%, and a 12-hour light/dark cycle. All the animals were allowed to adjust to the environment for a week before AP induction. All animal studies were reviewed and approved according to Ethics Committee of West China Hospital of Sichuan University.

### 2.2. CQCQD Preparation and Reagents

The Chinese medicinal herbs in CQCQD were purchased from the West China Hospital of Sichuan University (Chengdu, China). The detailed composition and preparation procedures were described in our previous work [21]. L-ornithine and carbachol were freshly prepared before each experiment using normal saline as the dissolving solvent. The concentration of L-ornithine stock was 30% (w/v), and its pH was adjusted to 7.0 with NaOH. IL-1*β* and TNF-*α* enzyme-linked immunosorbent assay (ELISA) kits were obtained from R&D (Minneapolis, MN, USA), while VIP and iFABP kits were from Cusabio Biotech (Wuhan, China). Antibodies against IL-1*β* (ab9722), TNF-*α* (ab11564), CPI-17 (ab322123), and phosphorylated-CPI-17 (p-CPI-17; ab52174) as well as fluorescence dyes FITC and TRITC were from Abcam (Cambridge, UK). Cy3 was from Molbase (Nanjing, China). Antibodies against p-MLC20 (3675S) and p-MYPT1 (5163S) were from Cell Signaling Technology (MA, USA). Fluo 4-AM was from Dojindo Laboratories (Minato-ku, Tokyo, Japan).

### 2.3. AP Model Induction and Interventions

Rats were randomly divided to 4 groups (*n* ≥ 4 per group) and received (1) 2 intraperitoneal injections of normal saline (3.0 g/kg) at 1 hour apart, (2) 2 intraperitoneal injections of L-ornithine (3.0 g/kg) at 1 hour apart [10, 31], L-ornithine injections and single intraperitoneal injection of CCh (60 *μ*g/kg) begun at 24 hours after the first L-ornithine injection, and (4) L-ornithine injections and 3 times oral gavage of CQCQD (20 g/kg) at 2 hourly interval begun at 24 hours after the first L-ornithine injection.

### 2.4. Sample Collection

Rats in all groups were humanly sacrificed at a range of time points after AP induction to assess disease severity. Blood samples were naturally clotted and centrifuged at 1500 g for 10 min to separate serum. The pancreas and the top part of the jejunum fragment were quickly removed and immersed into 10% formaldehyde solution for histopathology and immunofluorescence examination. The second and third part of jejunum fragments were also collected for western blotting and quantitative real-time polymerase chain reaction (RT-PCR), respectively. In separate experiments, the whole jejunum fragment was used to isolate SMCs and smooth muscle strips (SMS).

### 2.5. Serum Inflammatory and Indirect Intestinal Motility Biomarkers

Serum IL-1*β*, TNF-*α*, VIP, and iFABP levels were measured by ELISA kits according to manufacturer's instructions.

### 2.6. Histopathology

The formaldehyde-immersed samples were further embedded in the paraffin wax, sectioned into 5 mm slices, and stained with haematoxylin and eosin (H&E). After H&E staining, the pancreatic sections were scored according to oedema, inflammatory cell infiltration, and acinar cell necrosis [32]; the intestinal sections were scored following a previous protocol [33] with modification: the sum of severity of inflammation (none, slight, moderate, and severe), extension of inflammation (none, mucosa, mucosa and submucosa, and transmural), and crypt damage (none, basal 1/3 damaged, basal 2/3 damaged, and only surface epithelium intact). The scoring was done using 10 random visual fields (magnification 100x) by an experienced pathologist who was not aware of the study design.

### 2.7. Isolation of SMCs and SMS from Intestinal Smooth Muscle

A 10–15 cm jejunal segment was detached from its mesenteries and placed in sterile phosphate buffered saline (PBS) solution with 100 U/mL penicillin/streptomycin (1 : 1; pH 7.4) and peeled carefully off the mucosa, submucosa, and serosa. The isolation of jejunum SMCs followed our previous published protocol [21]. For SMS isolation, the jejunum fragment was quickly sheared and put into the Krebs–Henseleit solution with 100 U/mL penicillin/streptomycin for physiological property examination.

### 2.8. Contractility Assays

Jejunum SMS were quickly cut under 5 cm from pylorus for each group, approximately 2.5 cm in length. The SMS were placed in continually oxygenated (95% O_2_ and 5% CO_2_) and preheated (37°C) Kreb's solution (in mM: NaCl, 118.5; KCl, 4.8; KH_2_PO_4_, 1.2; MgSO_4_.7H_2_O, 1.2; CaCl_2_, 1.9; NaHCO_3_, 25; and glucose, 10.1 (pH 7.4)) and slightly removed the food residue. The SMS were longitudinally suspended under a 2 g load in the above conditions and slightly fixed to the two points by using the force-displacement transducer; make sure the solution can smoothly move through the bowel, then equilibration for 30 min. Tension generated along the longitudinal axis of the SMS was recorded by using an isometric tension transducer, and the activity of intestinal frequency value (cpm) and the tension value (g) was recorded for 15 mins using BL-420F biological data acquisition and analysis system (Chengdu Taimeng Software Co. LTD, China) [34, 35].

### 2.9. Immunofluorescence

The smears of SMS were immersed in the 10% formaldehyde solution for 15 mins and then in the 3% hydrogen peroxide solution for 15 mins. The slides were incubated for 5 mins in the 0.02 M PBS buffer (pH 7.4), blocked with the 5% bovine serum albumin Tris-HCl buffer at room temperature for 1 hour, incubated subsequently with the IL-1*β* (1 : 100), TNF-*α* (1 : 100), anti-CPI-17 (1 : 100), anti-p-CPI17 (1 : 100), anti-p-MLC20 (1 : 200), anti-p-MYPT1(1 : 200) for 2 hours at room temperature, and then washed in the PBS for 10 mins. Incubation was done with the secondary antibody with different fluorescence dyes: Cy3, FITC, and TRITC. The Envision System (DAKO, Copenhagen, Denmark) was used for visualisation of antibody binding. The diaminobenzidine was used as the chromogen for detection. All slides were then counterstained with haematoxylin, dehydrated, and mounted. The images were acquired using a Leica FV1000 laser scanning confocal microscope (Olympus, Tokyo, Japan) at the identical settings.

### 2.10. Measurement of [Ca^2+^]_i_

The details of [Ca^2+^]_i_ measurement in SMCs were described in our previous work [21]. Ten different cells in each visual field were randomly selected. The fluorescence of the Fluo 4-AM (final concentration: 7 *μ*mol/L) loaded cells was recorded using a Leica FV1000 laser scanning confocal microscope (Olympus, Tokyo, Japan). The relative fluorescence was analysed using fluorescence quantitative analysis software, and the intracellular Ca^2+^ fluorescence intensity was presented as [Ca^2+^]_i_.

### 2.11. RT-PCR and Western Blotting

The details of RT-PCR and western blotting procedures were reported in our previous publication [21]. Relative mRNA expression was normalised to *β*-actin level. Dilutions for primary antibody for western blotting were as follows: anti-IL-1*β* (1 : 300), anti-TNF-*α* (1 : 300), anti-CPI-17 (1 : 300), anti-p-CPI-17 (1 : 300), anti-p-MLC20 (1 : 500), and anti-p-MYPT1 (1 : 500). The protein of *β*-actin was used as internal housekeeping protein, and immunoreactivity was detected using a chemiluminescence's system and quantified by using ImageJ software (Bio-Rad, Hercules, USA) Table 1 shows the probe, primer, and product (bp) in RT-PCR.

### 2.12. Statistical Analysis

Data are expressed as means with standard errors of means (SEM). In all figures, vertical bars denote means ± SEM values. Statistical evaluation of the data was accomplished using a Student's *t*-test where data were normally distributed or otherwise a Mann–Whitney *U* test was adopted. The relative expression software tool was employed for statistical analysis of gene expression. Statistical analysis was performed using the statistical software package Origin 9.0 (OriginLab, Northampton, MA, USA), and a two-sided *P* value of <0.05 was considered to be significant.

## 3. Results

### 3.1. CQCQD Reduces L-Ornithine-Induced Necrotising AP and Systemic Inflammation

Representative pancreatic histopathology images (H&E) and summary scores are shown in Figures [Supplementary-material supplementary-material-1] and [Supplementary-material supplementary-material-1]. Saline injections did not induce significant histopathology changes of the pancreas; at 12 hours after the first L-ornithine injection, the overall pancreatic histopathology score begun to increase; at 24 hours, overt oedema, inflammatory cell infiltration, and acinar cell necrosis appeared and these were reflected by marked elevation of the individual and overall histopathology scores; at 36 and 48 hours, the histopathology changes and scores were similar to those at 24 hours but all were significantly higher than those at 12 hours or after saline injections ([Supplementary-material supplementary-material-1]). These pancreatic histopathology changes were in accord with previous published literature [21].

The effect of CQCQD and CCh on pancreatic and systemic injury was assessed at 30 hours after the first injection of L-ornithine ([Supplementary-material supplementary-material-1]). Both CQCQD and CCh significantly improved pancreatic histopathology and reduced overall histopathology score compared with L-ornithine injections alone. This was predominately attributed by the reduction of acinar cell necrosis. There was no significant reduction for oedema and inflammation scores. Furthermore, CQCQD markedly ameliorated the increased IL-1*β* and TNF-*α* levels caused by L-ornithine injections. Though there was a trend of reduction for these parameters after CCh application, statistical significance was not reached.

### 3.2. CQCQD Ameliorates L-Ornithine-Induced Gut Injury and Dysmotility

Representative jejunum histopathology images (H&E) and summary scores are shown in Figures 1 and 2. Similar to time-course pancreatic histopathological changes, the increase of jejunum histopathology changes and scores begun at 12 hours and thereafter (Figure 1(a)). At 12 hours, there were just scattered loss of villi, crypt damage, and mild inflammatory cell infiltration being demonstrated. These injuries became more apparent and were associated with marked crypt damage, increased inflammatory severity, and extent from 24 hours. These changes were mirrored by marked elevation of overall jejunum histopathology score at 24, 36, and 48 hours compared with 12 hours after the first L-ornithine injection or after saline injections (Figure 1(b)A). The patterns of breakdown scores were similar to the overall score, and at 36 and 48 hours, the crypt damage (Figure 1(b)B), inflammation severity (Figure 1(b)C), and extent (Figure 1(b)D) were the highest among all the time points.

The effect of CQCQD and CCh on jejunum injury and dysmotility was assessed at 30 hours after the first injection of L-ornithine. CQCQD significantly improved intestinal histopathology changes (Figure 2(a)) and dramatically reduced the overall intestinal histopathology score (Figure 2(b)A) which was mostly contributed by its profound effects on restricting crypt damage (Figure 2(b)B) and the extent of inflammation infiltration (Figure 2(b)D) compared with L-ornithine injections alone. Though CQCQD also appeared to reduce the severity of inflammation, there was no statistical significance reached (Figure 2(b)C). In addition, CQCQD significantly decreased serum VIP (Figure 2(c)) and iFABP (Figure 2(d)) levels, parameters that were elevated after L-ornithine injections and indirectly reflected gut dysmotility. In contrast to CQCQD, CCh did not significantly alter any of the intestinal histopathology and motility indices.

### 3.3. CQCQD Restores L-Ornithine-Induced Reduction of Jejunum SMC [Ca^2+^]_i_ and SMS Contractility

The representative images of isolated jejunum SMCs and [Ca^2+^]_i_ signals under confocal microscopy are displayed (Figure 3(a)). The morphological features of SMCs appeared to be oval, short spindle, or polygonal. L-ornithine caused reduction of [Ca^2+^]_i_ fluorescence intensity in SMCs to <25% of the controls at 24 and 30 hours after the first injection (both *P* < 0.05); this effect was significantly ameliorated in equal measure by the CCh or the CQCQD treatment (Figure 3(b)). The traces of resting-state contractility in each group were recorded by biological data acquisition and analysis system at 24 and 30 hours after the first L-ornithine injection (Figure 3(c)). There was significant reduction of both intestinal contractility tension (Figure 3(d)) and frequency (Figure 3(e)) under resting state compared with saline controls. The CQCQD treatment significantly enhanced both the intestinal contractility tension and frequency, while CCh only had significant effect on contractility tension.

### 3.4. CQCQD Counteracts L-Ornithine-Induced Increase of Inflammatory Cytokine Expression and Decrease of CPI-17 Expression in Jejunum SMS

Example images of agarose gel electrophoresis after RT-PCR for mRNA of IL-1*β*, TNF-*α*, CPI-17, and *β*-actin in SMS collected at 24 and 30 hours after the first L-ornithine injection are shown (Figure 4(a)). L-ornithine caused significant elevation of IL-1*β* and TNF-*α* as well as reduction of CPI-17 (Figure 4(b)). Both CQCQD and CCh treatments significantly reduced IL-1*β* mRNA expression and increased CPI-17 mRNA expression compared with L-ornithine injections alone at 30 hours. Though there was an apparent reduction of TNF-*α* mRNA expression after CQCQD or CCh treatment, none of them reached statistical significance.

Example images of agarose gel electrophoresis after western blotting for IL-1*β*, TNF-*α*, CPI-17, and *β*-actin in SMS collected at 24 and 30 hours after the first L-ornithine injection are shown (Figure 4(c)). The changes of protein expression were similar to what were observed for these mRNAs (Figure 4(d)). Both CQCQD and CCh treatments significantly decreased IL-1*β* protein expression and increased CPI-17 protein expression compared with L-ornithine injections alone at 30 hours. Though CCh was shown to reduce TNF-*α* protein expression, there was no significant reduction after CQCQD treatment. Illustrative fluorescence images of IL-1*β*, TNF-*α*, and CPI-17 in SMS are also demonstrated (Figure 4(e)), reflecting similar findings to RT-RCR and western blotting analyses.

### 3.5. CQCQD Prevents L-Ornithine-Induced Reduction of Phosphorylated CPI-17, MYPT1, and MLC20 in Jejunum SMS

We observed an increase of MYPT1 expression at both 24 and 30 hours after L-ornithine administration when compared with the control group; CCh but not CQCQD significantly reduced the MYPT1 expression ([Supplementary-material supplementary-material-1]). The representative western blot images (Figure 5(a)) show there was consistently and significantly decreased phosphorylation of CPI-17, MYPT1, and MLC20 expression at 30 hours after L-ornithine administration (Figure 5(b)). Both CQCQD and CCh treatments significantly prevented L-ornithine-induced reduction of protein phosphorylation, with the greatest magnitude associated with the CQCQD. Phosphorylated CPI-17, MYPT1, and MLC20 were observed in smooth muscle layer, submucosa, and mucosa by immunofluorescence staining. Similarly, in smooth muscle layer, phosphorylation of CPI-17, MYPT1, and MLC20 expression at 30 hours after L-ornithine administration was decreased. Both CQCQD and CCh treatments increased the fluorescence intensity detected by confocal microscopy (Figure 5(c)).

### 3.6. Summary of the Role of CQCQD in Early Stage of AP

As shown in Figure 6, the CQCQD has been approved to (1) reduce cytokines (e.g., IL-1*β* and TNF-*α*), neurotransmitters (e.g., substance P and VIP) that are released from the injured pancreas and residential immune cells to improve AP and (2) alleviate gut injury and improve gut motility at least in part via modulating the CPI-17/MLCP pathway in SMS.

## 4. Discussion

Ileus is the most frequent complication in AP patients. Improvement of gastrointestinal dysmotility timely was contributed to the prognosis of AP. Recent clinical trials have indicated that rhubarb [36] and CQCQD derivatives [37–40] reduce intra-abdominal pressure, shorten the duration of ileus, and improve clinical outcomes. However, the mechanism is unknown. This is the first study that characterised the time-course histopathological changes of gut injury and dysmotility in L-ornithine-induced necrotising AP in rats. L-ornithine-induced pancreatic acinar cell necrosis and inflammation were associated with marked elevation of systemic injury biomarkers (serum IL-1*β* and TNF-*α*) and gut injury and altered indirect gut motility parameters (serum VIP and iFABP). We found L-ornithine-induced gut dysmotility can be partially explained by decreased intestinal smooth muscle contractility that was regulated by the Ca^2+^ sensitisation-mediated deranged CPI17/MLCP pathway. Both CQCQD and CCh alleviated these effects caused by L-ornithine and improved gut motility, and CQCQD was more effective than CCh.

The gastrointestinal tract is one of the most easily damaged organs in the development of AP, and gut injury and gut dysmotility also contribute to the severity of AP [1–3]. It is generally known that inflammatory cytokines play a critical role in gut injury and dysmotility [15]. On the other hand, severe AP is associated with a local and systemic overproduction of inflammatory cytokines [20], especially IL-1*β* and TNF-*α* which can activate macrophages in the intestine and result in intestinal injury, dysmotility, and increased permeability [18, 19]. Subsequently, the absorption of endotoxin and overgrowth and translocation of bacteria in the intestine result in systemic inflammation and MODS [3]. Thus, a “gut-centred” therapeutic strategy has been recognised as important in the early management of AP [41]. This approach has been developed in West China Hospital over the past thirty years through using an integrated approach that combines traditional Chinese (such as the CQCQD mixture and its derivatives or a single component treatment, e.g., rhubarb) and standard Western medicine approaches [42, 43]. Both clinical and experimental studies have now clearly demonstrated that an integrated approach can improve adverse clinical outcomes, including a reduction in gut dysmotility [21, 38, 40], respiratory failure [44, 45], and proinflammatory cytokines [46, 47].

In this study, it was shown that L-ornithine induced intestinal damage as shown by the increase of the serum VIP, and iFABP levels, and was consistent with our previous study [21]. The marker VIP is widely used as an indirect parameter for gut motility assessment, and its increase is associated with underlying gut dysmotility in experimental and human AP [5, 40]. iFABP is a sensitive biomarker for the detection of intestinal injury, and its increased levels are correlated with AP severity in patients [48]. CQCQD significantly reduced L-ornithine-induced increases of VIP and iFABP, returning them towards the normal range. The improvement for gut motility and AP severity is consistent with what has been reported with the CQCQD (and its derivatives) treatment in other AP models [21] and AP patients [40]. CCh showed a trend to decrease the serum VIP and iFABP in L-ornithine-induced AP, indicating its potential role in the protection of gut motility.

The available evidence suggests that CPI-17 plays a pivot role in inflammation-induced gut dysmotility [27]. CPI-17 is an endogenous inhibitor of serine/threonine protein phosphatase in SMCs, and activation of CPI-17 mediates Ca^2+^-independent sustained contraction induced by various agonists in SMCs [24, 49]. It has been shown that downregulation of CPI-17 expression appeared in TNBS-induced and dextran sodium sulphate-induced ulcerative colitis animal models [50, 51] and also in patients [52]. Thus, CPI-17 downregulation during gut inflammation is associated with the decreased contractile response of inflamed smooth muscle, and plenty of inflammatory cytokines contribute to this pathophysiological process. IL-1*β* and TNF-*α* are proinflammatory cytokines that can block the contraction of gut SMCs [53, 54] and have been shown to be increased in intestinal mucus in AP models [55, 56]. IL-1*β* can upregulate RGS4 expression, which not only results in the inhibition of the initial contraction through inhibiting PLC-*β* activation but also downregulates CPI-17 expression, and subsequently suppresses CPI-17 phosphorylation to inhibit MLCP, and finally, leads to the inhibition of sustained MLC20 phosphorylation and muscle contraction [29]. It is well documented that IL-1*β* decreases CPI-17 activity and gut smooth muscle contraction through generating TNF-*α* and CPI-17 downregulation appears after IL-1*β*-induced TNF-*α* production [28]. In this study, we observed upregulation of IL-1*β* and TNF-*α* expression and downregulation of CPI-17 expression in L-ornithine-induced AP as well as decrease of smooth muscle contractility. In consistent with our previous study, the increased IL-1*β* and TNF-*α* expression appeared earlier than decreased CPI-17 expression. In our study, we investigated that CQCQD and CCh treatment significantly decreased the IL-1*β* expression and increased the CPI-17 expression in L-ornithine-induced AP. The CCh treatment significantly decreased the TNF-*α* protein expression, while CQCQD only had minor effects. The reason may be that, *in vivo*, many other cytokines may contribute to the induction of TNF-*α*, and elevation of TNF-*α* appeared within 3 hours after AP onset in the superior mesenteric vein [55]. However, in our study, CQCQD was administered only at 24 hours after AP onset. Further studies are needed to assess the effect of early administration of CQCQD in modulating IL-1*β* and TNF-*α* in SMS.

Synchronous phosphorylation sites in CPI-17 and MYPT1 play essential roles in sustained MLC20 phosphorylation and force greater development at a given [Ca^2+^]_i_; thus, this process leads to intestinal smooth muscle contraction [15, 57, 58]. Our study was consistent with this mechanism. We observed that the intestinal contraction decreased by reduction of MLC20 phosphorylation through decreased phosphorylation of CPI-17 and MYPT1 of intestinal SMS in L-ornithine-induced AP rats. Our previous study indicated that both CQCQD and CCh increased initial intestinal contraction via the PLC-*β* and PKC pathway by increasing [Ca^2+^]_i_ of colonic SMCs in L-arginine-induced AP rats [21]. In this study, both CQCQD and CCh significantly increased the synchronous phosphorylation of CPI-17 at thr^38^ and MYPT1 at Thr^696^ in SMS and the elevation of [Ca^2+^]_i_ in SMCs, leading to phosphorylation of MLC20, thus improving intestinal motility and pancreatic histopathology. These findings indicate that impairment of the Ca^2+^-sensitivity pathway, especially the CPI-17/MLCP pathway in intestinal smooth muscle played a role in the pathogenesis of intestinal dysmotility in experimental AP. It is generally known that CCh increases [Ca^2+^]_i_ through the G protein pathway to induce contraction in intestinal smooth muscles. *In vitro*, CCh-induced intestinal contraction was also through the Ca^2+^-independent pathway, by increasing phosphorylation of CPI-17 and MYPT1 [57]. This process, however, is inhibited by IL-1*β* and TNF-*α*. Thus, at least, the molecular mechanism of improving intestinal contraction by CQCQD in experimental AP is indirectly explained.

## 5. Conclusions

Gut injury and dysmotility are found in severe clinical AP and were shown here to be also present in L-ornithine-induced necrotising AP in rats. Both CQCQD and CCh in this model tended to decrease inflammatory cytokines of intestinal smooth muscle, improve gut motility, and attenuate the overall severity of necrotising AP. This beneficial effect on gut motility may result from modulating the CPI-17/MLCP pathway in intestinal smooth muscles by reducing proinflammatory cytokines.

## Figures and Tables

**Figure 1:** Time-course intestinal histopathology changes in L-ornithine-induced acute necrotising pancreatitis. Rats received 2 intraperitoneal injections of L-ornithine (Orn; 3.0 g/kg; pH 7.0) at 1 hour apart and controls received the same regimen of normal saline injections. Rats were sacrificed at 12, 24, 36, and 48 hours to assess severity of acute pancreatitis. (a) Representative H&E sections of upper jejunum (100x). (b) Intestinal histopathology scores: A, overall; B, crypt damage; C, inflammation severity; D, inflammation extent. ^*∗*^*P* < 0.05*vs.* saline group; ^†^*P* < 0.05*vs.* L-ornithine 12 h group. Values are means ± SEM of 4–6 animals per group.

**Figure 2:** Effects of CQCQD and CCh on intestinal histopathology and serum intestinal motility biomarkers. Rats received 2 intraperitoneal injections of L-ornithine (Orn; 3.0 g/kg; pH 7.0) at 1 hour apart and controls received the same regimen of normal saline injections. In the treatment groups, rats either received single intraperitoneal injection of carbachol (CCh; 60 *μ*g/kg) or 3 times oral gavage of chaiqin chengqi decoction (CQCQD; 20 g/kg) at 2-hourly interval begun at 24 hours after the first L-ornithine injection. Rats were sacrificed at 30 hours to assess severity of acute pancreatitis. (a) Representative H&E sections of upper jejunum (100x). (b) Intestinal pathology scores: A, overall; B, crypt damage; C, inflammation severity; D, inflammation extent. (c) Serum vasoactive intestinal peptide (VIP). (d) Serum intestinal fatty acid-binding protein (iFABP). ^*∗*^*P* < 0.05*vs.* saline group; ^†^*P* < 0.05*vs.* L-ornithine group. Values are means ± SEM of 5–10 animals per group.

**Figure 3:** Effects of CQCQD and CCh on [Ca^2+^]_i_ in cells and contraction in strips of jejunum smooth muscles. Rats received 2 intraperitoneal injections of L-ornithine (Orn; 3.0 g/kg; pH 7.0) at 1 hour apart and controls received the same regimen of normal saline injections. In the treatment groups, rats either received single intraperitoneal injection of carbachol (CCh; 60 *μ*g/kg) or 3 times oral gavage of chaiqin chengqi decoction (CQCQD; 20 g/kg) at 2-hourly interval begun at 24 hours after the first L-ornithine injection. Rats were sacrificed at 24 or 30 hours to isolate jejunum smooth muscle cell and strips for assessing intracellular calcium concentrations [Ca^2+^]_i_ and contraction, respectively. (a) Representative confocal microscopy images of Fluo 4-AM stained (×200). The lower left corner for each image is a representative morphological observation field of isolated smooth muscle cell (200x). (b) Fluo 4-AM fluorescence intensity (FI) for all experimental groups. (c) Example images of jejunum smooth muscle strip contraction for each experimental group. *X* axis represents time in seconds and *Y* axis represents (g) (d) Contraction tension. (e) Contraction frequency. All data are normalised according to saline injection group using arbitrary unit (AU). The bar of medium and sparse patterns represents rats sacrificed at 24 and 30 hours after the first L-ornithine/saline injection, respectively. ^*∗*^*P* < 0.05*vs.* saline group; ^†^*P* < 0.05*vs.* L-ornithine group. Values are means ± SEM of 4 animals per group.

**Figure 4:** Effects of CQCQD and CCh on mRNA and protein expression of IL-1*β*, TNF-*α*, and CPI-17 in jejunum smooth muscle strips. Rats received 2 intraperitoneal injections of L-ornithine (Orn; 3.0 g/kg; pH 7.0) at 1 hour apart and controls received the same regimen of normal saline injections. In the treatment groups, rats either received single intraperitoneal injection of carbachol (CCh; 60 *μ*g/kg) or 3 times oral gavage of chaiqin chengqi decoction (CQCQD; 20 g/kg) at 2-hourly interval begun at 24 hours after the first L-ornithine injection. Rats were sacrificed at 24 or 30 hours to isolate jejunum smooth muscle strips. (a) Representative images of agarose gel electrophoresis of targeted RT-PCR mRNAs. (b) Histograms for semiquantitative mRNA expression. (c) Representative western-blotting images of proteins. (d) Histograms for semiquantitative protein expression. (e) Example images of immunofluorescence (s, smooth muscle layer; m, mucosa; sm, submucosa). Relative expression of individual mRNA and protein are calculated according to *β*-actin. The bar of medium and sparse patterns represents rats sacrificed at 24 and 30 hours after the first L-ornithine/saline injection, respectively. ^*∗*^*P* < 0.05*vs.* saline group, ^†^*P* < 0.05*vs.* L-ornithine group; ^‡^*P* < 0.05*vs.* CCh-treated group. Values are means ± SEM of 4 animals per group.

**Figure 5:** Effects of CQCQD and CCh on mRNA and protein expression of p-CPI-17, p-MYPT1, and p-MLC20 in jejunum smooth muscle strips. Rats received 2 intraperitoneal injections of L-ornithine (Orn; 3.0 g/kg; pH 7.0) at 1 hour apart and controls received the same regimen of normal saline injections. In the treatment groups, rats either received single intraperitoneal injection of carbachol (CCh; 60 *μ*g/kg) or 3 times oral gavage of chaiqin chengqi decoction (CQCQD; 20 g/kg) at 2-hourly interval begun at 24 hours after the first L-ornithine injection. Rats were sacrificed at 24 or 30 hours to isolate jejunum smooth muscle strips. (a) Representative images of agarose gel electrophoresis of targeted RT-PCR mRNAs. (b) Histograms for semiquantitative mRNA expression. (c) Representative western-blotting images of proteins. (d) Histograms for semiquantitative protein expression. (e) Example images of immunofluorescence (s, smooth muscle layer; m, mucosa; sm, submucosa). ^*∗*^*P* < 0.05*vs.* saline group, ^†^*P* < 0.05*vs.* L-ornithine group, and ^‡^*P* < 0.05*vs.* CCh-treated group. Values are means ± SEM of 4 animals per group.

**Figure 6:** Summary diagram of the role of CQCQD in early stage of acute pancreatitis. SIRS, systemic inflammatory response syndrome; MODS, multiple organ dysfunction syndrome.

**Table 1:** Probe, primer, and product (*bp*) in RT-PCR.

Gene	Forward and reverse primer pair sequences	Annealing temperature (°C)	Primer bases (bp)
IL-1*β*	F : CAACAAGTGGTATTCTCCAT	52	177
	R : TTCCATCTTCTTCTTTGGGT		
	TM : CCTGTGGCCTTGGGCCTC		
TNF-*α*	F : CACGTCGTAGCAAACCACCAA	54	100
	R : GTTGGTTGTCTTTGAGATCCAT		
	TM : CCACTCCAGCTGCTCCTCC		
CPI-17	F : GGCTGCAGAAGCGGCAC	58	129
	R : GCATGTCTGCCTCCCTGC		
	TM : CTGGACGTGGAGAAGTGGATC		
*β*-Actin	F : GAAGATCAAGATCATTGCTCCT	52	111
	R : TACTCCTGCTTGCTGATCCACA		
	TM : TCACTGTCCACCTTCCAGCAGA		

## Data Availability

The data used to support the findings of this study are available from the corresponding author upon request.

## Supplementary Materials

Supplementary Materials Figure S1: time-course pancreatic histopathology changes in L-ornithine-induced acute necrotising pancreatitis. Rats received 2 intraperitoneal injections of L-ornithine (Orn; 3.0 g/kg; pH 7.0) at 1 hour apart and controls received the same regimen of normal saline injections. Rats were sacrificed at 12, 24, 36, and 48 hours to assess severity of acute pancreatitis. (a) Representative H&E sections of pancreatic head (×100). (b) Pancreatic histopathology scores: A, overall; B, oedema; C, inflammation cell infiltration; D, acinar cell necrosis. ^*∗*^*P* < 0.05 vs. saline injection group; ^†^*P* < 0.05 vs. L-ornithine 12 h group. Values are means ± SEM of 4–6 animals per group. Figure S2: effects of CQCQD and CCh on pancreatic histopathology and serum proinflammatory biomarkers. Rats received 2 intraperitoneal injections of L-ornithine (Orn; 3.0 g/kg; pH 7.0) at 1 hour apart and controls received the same regimen of normal saline injections. In the treatment groups, rats either received single intraperitoneal injection of carbachol (CCh; 60 *μ*g/kg) or 3 times oral gavage of chaiqin chengqi decoction (CQCQD; 20 g/kg) at 2-hourly interval begun at 24 hours after the first L-ornithine injection. Rats were sacrificed at 30 hours to assess severity of acute pancreatitis. (a) Representative H&E sections of pancreatic head (×100). (b) Pancreatic histopathology scores: A, overall; B, oedema; C, inflammatory cell infiltration; D, acinar cell necrosis. (c) Serum interleukin-1beta (IL-1â). (d) Serum tumour necrosis factor-alpha (TNF-á). ^*∗*^*P* < 0.05 vs. saline group; ^†^*P* < 0.05 vs. L-ornithine group. Values are means ± SEM of 5–10 animals per group. Figure S3: effects of CQCQD and CCh on protein expression of MYPT1 in jejunum smooth muscle strips. Rats received 2 intraperitoneal injections of L-ornithine (Orn; 3.0 g/kg; pH 7.0) at 1 hour apart and controls received the same regimen of normal saline injections. In the treatment groups, rats either received single intraperitoneal injection of carbachol (CCh; 60 ìg/kg) or 3 times oral gavage of chaiqin chengqi decoction (CQCQD; 20 g/kg) at 2-hourly interval begun at 24 hours after the first L-ornithine injection. Rats were sacrificed at 24 or 30 hours to isolate jejunum smooth muscle strips. (a) Representative western-blotting images of proteins. (b) Histograms for semiquantitative protein expression. ^*∗*^*P* < 0.05 vs. saline group; ^†^*P* < 0.05 vs. L-ornithine group. Values are means ± SEM of 4 animals per group.
